This article has been retracted.

# P38 and ERK1/2 MAPKs Act in Opposition to Regulate BMP9-Induced Osteogenic Differentiation of Mesenchymal Progenitor Cells

**DOI:** 10.1371/journal.pone.0043383

**Published:** 2012-08-17

**Authors:** Yingze Zhao, Tao Song, Wenjuan Wang, Jin Wang, Juanwen He, Ningning Wu, Min Tang, Baicheng He, Jinyong Luo

**Affiliations:** Key Laboratory of Diagnostic Medicine designated by the Chinese Ministry of Education, Chongqing Medical University, Chongqing, China; University of South Florida College of Medicine, United States of America

## Abstract

Although previous studies have demonstrated that BMP9 is highly capable of inducing osteogenic differentiation and bone formation, the precise molecular mechanism involved remains to be fully elucidated. In this current study, we explore the possible involvement and detail effects of p38 and ERK1/2 MAPKs on BMP9-indcued osteogenic differentiation of mesenchymal progenitor cell (MPCs). We find that BMP9 simultaneously stimulates the activation of p38 and ERK1/2 in MPCs. BMP9-induced early osteogenic marker, such as alkaline phosphatase (ALP), and late osteogenic markers, such as matrix mineralization and osteocalcin (OC) are inhibited by p38 inhibitor SB203580, whereas enhanced by ERK1/2 inhibitor PD98059. BMP9-induced activation of Runx2 and Smads signaling are reduced by SB203580, and yet increased by PD98059 in MPCs. The *in vitro* effects of inhibitors are reproduced with adenoviruses expressing siRNA targeted p38 and ERK1/2, respectively. Using mouse calvarial organ culture and subcutaneous MPCs implantation, we find that inhibition of p38 activity leads to significant decrease in BMP9-induced osteogenic differentiation and bone formation, however, blockage of ERK1/2 results in effective increase in BMP9-indcued osteogenic differentiation *in vivo*. Together, our results reveal that p38 and ERK1/2 MAPKs are activated in BMP9-induced osteogenic differentiation of MPCs. What is most noteworthy, however, is that p38 and ERK1/2 act in opposition to regulate BMP9-induced osteogenic differentiation of MPCs.

## Introduction

Mesenchymal progenitor cells (MPCs) are non-hematopoietic stem cells capable of differentiating into osteoblastic, chondrogenic, myogenic, or adipogenic lineages [1], [2], [3], [4], [5]. Although recent studies have demonstrated that MPCs are also able to differentiate into other lineages, including neuronal and cardiomyogenic lineages [6], [7], [8]. Bone morphogenetic proteins (BMPs), members of transforming growth factors beta (TGFβ) superfamily, are known to play important roles in stem cell biology and perform pivotal functions in the areas of embryogenesis, multiple growth and differentiation processes [9], [10], [11], [12]. Genetic disruptions of BMPs have led to various skeletal and extra-skeletal abnormalities during development [9], [13]. To date, more than twenty BMPs have been identified. Several forms of recombinant BMPs, most notably BMP2 and BMP7, have been shown to promote osteogenesis and are now used as adjunctive therapy in the clinical setting [14], [15], [16], [17], [18]. However, it remains unclear whether BMP2 and BMP7 are in fact the most potent BMPs in inducing osteogenic differentiation and bone formation.

Recent studies have implied us that BMP9, one of the least studied BMPs, is probably a more potent inducer in promoting osteogenic differentiation of MPCs *in vitro* and *in vivo* [11], [19], [20], [21]. Furthermore, a distinct set of downstream target genes that may play a role in regulating BMP9-induced osteogenic differentiation of MPCs were identified by microarray [11], [20]. Our recent study revealed that TGFβ type I receptors ALK1 and ALK2 are essential for BMP9-induced osteogenic signaling in MPCs [22]. We also elucidated that TGFβ type II receptors BMPRII and ActRII are the functional receptors necessary to transmit osteoinductive signaling of BMP9 [23]. Despite these valuable discoveries, BMP9 remains as the least characterized BMPs, and the signaling mechanism through which BMP9 regulates osteogenic differentiation of MPCs is still largely unknown and warrants extensive studies.

It has been well established that BMPs fulfill their signaling activity through activation of transcription factors Smads. In this case, BMPs signal transduction begins with binding to heterodimeric complex of two transmembrane serine/threonine kinase receptors, BMPs type I and type II receptors [9], [10], [22], [23]. These activated receptors transmit signals by phosphorylating the transcription factors Smads (Smad1, 5, and/or 8) [9], [10], [22], [23], [24], [25], [26], which in turn form a heterodimeric complex with Smad4 in the nucleus and modulate context-dependent gene expression in collaboration with other co-activators. However, growing evidences have implied that BMPs also utilize diverse intracellular signaling molecules in addition to Smads to regulate a wide array of cellular functions [26], [27], [28], [29], [30], [31], [32], [33], [34], [35], [36], [37], [38], [39], [40], [41], [42], [43], [44], [45]. These are collectively called the non-Smads (non-canonical) pathway of BMPs signaling. Mitogen activated protein kinases (MAPKs), such as p38 and extracellular signal-regulated kinase (ERK1/2), are key branch of non-Smads BMPs pathway [26], [27], [28], [29], [30], [31], [32], [33], [34], [35], [36], [37], [38], [39], [40], [41], [42].

MAPKs are a group of well-described serine/threonine-specific protein kinases generally expressed in all cell types [46], [47], [48]. At least four subfamilies of mammalian MAPKs have been identified, including ERK1/2, ERK5 (also known as MAPK7 or BMK1), the Jun amino-terminal kinases (JNKs) and p38 MAPKs. Each class of MAPKs is activated by a distinct kinase cascade in which a MEKK phosphorylates and stimulates a downstream dual-specificity MEK, which in turn phosphorylates threonine/tyrosine residues on MAPKs. Phosphorylation of these threonine/tyrosine residues on MAPKs results in a conformational change that evokes MAPKs activity [49]. MAPKs are essential components of signal transduction machinery and occupy a central position in regulation of gene expression, mitosis, metabolism, survival, motility, apoptosis, proliferation and differentiation [47], [50], [51], [52]. However, the different MAPKs members are activated in response to different extracellular stimuli and have different downstream targets, and thus play distinct roles in cellular responses.

Although it has been demonstrated that BMP9 plays a critical role in the processes by which MPCs undergo commitment to the osteoblastic lineage, little is known about the downstream signaling pathway(s) involved. In our previous studies, we have found that BMP9 is capable of simulating the expression of Smad6 and Smad7 (early targets of BMPs-Smads signaling) [22], [23]. Moreover, we further demonstrated that BMP9 is able to increase Smad1/5/8 transcriptional activity and enhance translocation of Smad1/5/8 to the nucleus in MPCs [22], [23], [24]. In another study by Bergeron *et al*., BMP9 was found to fulfill osteoinductive effects on MC3T3-E1 preosteoblastic cells by phosphorylating downstream Smads transcriptional factors [25]. These reports intensively validate that BMP9 can induce osteogensis and bone formation through activation of the Smads signaling pathway. However, the non-Smads pathways in BMP9-induced osteogenesis are largely unknown and need to be intensively explored.

It has been well demonstrated that MAPKs play a critical role in transmitting intracellular signaling of osteoinductive BMPs, such as BMP2 and BMP4, in MPCs [34], [35], [36], [37], [38], [39], [40], [41], [42]. However, whether MAPKs are also relevant to BMP9-induced osteogenic differentiation of MPCs are currently unclear. In the present study, we try to probe the possible involvement and exact function of two classic MAPKs subfamilies, p38 and ERK1/2 in regulating BMP9-indcued osteogenic differentiation of MPCs. Our results show that p38 and ERK1/2 MAPKs are both activated by BMP9 treatment in MPCs. Inhibition of p38 by specific inhibitor SB203580 or RNAi dramatically reduces BMP9-indcued osteogenic differentiation and Smads signaling *in vitro*, decreases BMP9-induced bone formation *in vivo*. Conversely, blocking of ERK1/2 by specific inhibitor PD98059 or RNAi enhances BMP9-induced osteogenic differentiation and Smads signaling, and increases BMP9-induced bone formation. Taken together, these results strongly suggest that BMP9 can simultaneously stimulate phosphorylation/activation of p38 and ERK1/2 MAPKs. Also, it’s important to note that p38 and ERK1/2 MAPKs are probably to act in opposition to regulate BMP9-induced osteogenic differentiation of MPCs.

## Materials and Methods

### Cell Culture and Chemicals

C3H10T1/2, C2C12, HEK293 and HCT116 cell lines were obtained from ATCC (American Type Culture Collection, Manassas, VA)and maintained in complete DMEM medium supplemented with 10% fetal calf serum (FCS, Hyclone) and antibiotics. MAPKs inhibitors PD98059 and SB203580 were obtained from Santa Cruz Biotechnology (California, USA). Inhibitors were dissolved in DMSO and aliquots were stored in −80°C. Unless indicated otherwise, all chemicals were purchased from Sigma-Aldrich (Saint Louis, USA).

### Isolation of Mouse Embryo Fibroblasts (MEFs)

MEFs were isolated from post coitus day 13.5 mice, as previously described [22], [23]. Briefly, each embryo was dissected into 10 ml sterile PBS, voided of its internal organs, and sheared through an 18-gauge syringe in the presence of 1 ml 0.25% trypsin and 1 mM EDTA. After 15 min incubation with gentle shaking at 37°C, DMEM with 10% FCS was added to inactivate trypsin. The cells were plated on 100 mm dishes and incubated for 24 hr at 37°C. Adherent cells were used as MEFs. Aliquots were kept in a liquid nitrogen tank. All MEFs used in this study were less than five passages.

### Construction of Recombinant Adenoviruses

Recombinant adenoviruses expressing BMP9 (Ad-BMP9) were generated previously using the AdEasy system, as demonstrated [21], [22], [23], [24]. Recombinant adenoviruses expressing small interference RNA (siRNA) targeted p38 (AdR-si-p38), ERK1/2 (AdR-si-ERK1/2) were kindly provided by Dr. Tong-chuan He of University of Chicago Medical Center. Adenoviruses expressing only GFP (Ad-GFP) and RFP (Ad-RFP) were used as controls.

### Preparation of Conditioned Medium

BMP9 conditioned media (BMP9-CM) were prepared as described [22], [23]. Briefly, subconfluent HCT116 cells (in 75-cm2 flaks) were infected with an optimal titer of Ad-BMP9. At 24 hrs after infection, the culture medium was changed to serum-free DMEM. Conditioned medium was collected at 48 hrs after infection and used immediately.

### Western Blotting Analysis

Briefly, cells were collected and lysed in RAPI buffer. Cleared total cell lysate was denatured by boiling and loaded onto a 10% gradient SDS–PAGE. After electrophoretic separation, proteins were transferred to an Immobilon-P membrane. Membrane was blocked with Super-Block Blocking Buffer, and probed with the primary antibody, followed by incubation with a secondary antibody conjugated with horseradish peroxidase. The proteins of interest were detected by using SuperSignal West Pico Chemiluminescent Substrate kit. Primary antibodies were obtained from Santa Cruz, as follows: anti-phosphor-p38, anti-p38, anti-phosphor-ERK1/2, anti-ERK1/2, anti-phosphor-Smad1/5/8, anti-Smad1/5/8, anti-Runx2 and anti-β-actin.

### Alkaline Phosphatase (ALP) Assays

ALP activity was assessed by a modified Great Escape SEAP Chemiluminescence assay (BD Clontech, Mountain View, CA), as described previously [19], [20], [21], [22], [23]. Each assay condition was performed in triplicate and the results were repeated in at least three independent experiments. ALP activity was normalized by total cellular protein concentrations among the samples.

### Matrix Mineralization Assay

Cultured cells were seeded in 24-well cell culture plates and infected with Ad-BMP9 followed by treated with PD98059 or SB203580, or infected with AdR-si-p38 (or AdR-si-ERK1/2) followed by treat with BMP9-CM. Cells were cultured in the presence of ascorbic acid (50 µg/ml) and β-glycerophosphate (10 mM). At 21 days after cultured, mineralized matrix nodules were stained for calcium precipitation by means of Alizarin Red S staining, as described previously [21], [22], [23]. Briefly, cells were fixed with 0.05% (v/v) glutaraldehyde at room temperature for 10 min. After being washed with distilled water, fixed cells were incubated with 0.4% Alizarin Red S (Sigma-Aldrich) for 5 min, followed by extensive washing with distilled water. The staining of calcium mineral deposits was recorded under bright field microscopy.

### Immunocytochemical Stain

Cultured cells were infected with Ad-BMP9 or Ad-GFP followed by treated with PD98059 and SB203580, or infected with AdR-si-p38 (or AdR-si-ERK1/2) and followed by BMP9-CM treatment. At the indicated time points, cells were fixed with 4% formalin and washed with PBS. The fixed cells were permeabilized with 0.25% Triton X-100 and blocked with 10% goat serum, followed by incubation with an anti-osteocalcin antibody (Santa Cruz Biotechnology) overnight. After washing, cells were incubated with biotin-labeled secondary antibody for 30 min, followed by incubating cells with streptavidin-HRP conjugate for 20 min at room temperature. The presence of the expected protein was visualized by DAB staining and examined under a microscope. Stains without the primary antibody, or with control IgG, were used as negative controls.

### Immunofluorescence Staining

Cultured cells were treated with PD98059 and SB203580 followed by stimulated with BMP9-CM. At the indicated time points, cells were fixed with 4% formalin and washed with PBS. The fixed cells were permeabilized with 0.25% TriTon X-100, followed by incubation with a polyclone anti-Smad1/5/8 antibody (Santa Cruz Biotechnology) overnight. After washing, cells were incubated with FITC fluorescein conjugated secondary antibody for 30 min. Fluorescence signal was recorded under a fluorescence microscope.

### RNA Isolation and Quantitative Real-time RT-PCR (qPCR)

Total RNA was extracted from cells with Trizol reagents (Invitrogen), and was used to generate cDNA by hexamer (Takara) and MMLV reverse transcriptase (Promega, CA, USA). PCR primers (**Table S1**) were designed by using the Primer3 program. SYBR Green-based qPCR analysis was carried out to amplify the genes of interest using RG-3000 Real-Time DNA Detection System (Corbett Research, Australia). Triplicate reactions were carried out for each sample. The cycling program was as: 94°C for 2 min for 1 cycle and 30 cycles at 92°C for 20 s, 57°C for 30 s, and 72°C for 20 s, followed by a plate read at 78°C for each cycle. All samples were run in triplicate and normalized by the endogenous expression level of β-actin.

### Subcutaneous MPCs Implantation

All animal experiments were approved by Institutional Animal Care and Use Committee (IACUC) of Chongqing Medical University. The ectopic bone formation by MPCs implantation was conducted as described [22], [23,23]. C3H10T1/2 cells were co-infected with Ad-BMP9 and Ad-si-p38 (or Ad-si-ERK1/2). Cells were collected at 80% confluence and for subcutaneous injection (5×10^6^/injection) into the flanks of athymic nude mice (6 animals per group, 4–6-week old, male, Harlan Sprague Dawley). At 5 weeks after implantation, animals were killed, and the implantation sites were retrieved for histological stains, as follows: Retrieved tissues were decalcified, fixed in 10% formalin overnight, and embedded in paraffin. Serial sections of the embedded specimens were stained with hematoxylin and eosin (H&E) stain. Masson’s Trichrome stain was carried out as described [22], [23]. Deparaffinized and rehydrated sections were stained with 1% Alcian Blue (pH 2.5), as described previously [22], [23].

### Mouse Calvarial Organ Culture

Calvariae was isolated from 4 days old mouse pulps, and culture in media containing BMP9 and SB203580 (or PD98059) for 4 days. Then, the calvariae was placed into fresh media and return to incubator for another 3 day until day 7. The hematoxylin and eosin staining (H&E staining) was conducted to measure the total area of original bone remaining. In H&E staining, the eosin Y differentially stains the original bone darker whereas the new bone matrix that is formed appears as a lighter color [53]. The width of new bone was determined by Image Pro Plus.

## Results

### BMP9 Stimulates Phosphorylation/activation of p38 and ERK1/2 MAPKs in MPCs

First of all, we sought to determine if p38 and ERK1/2 MAPKs can be activated by BMP9 in MPCs. Proliferating C3H10T1/2 cells were infected with Ad-BMP9 or Ad-GFP, then phosphorylation of Smad1/5/8, p38 and ERK1/2 were assessed by western blotting. Consistent with the results from pervious reports [22], [23], [24], [25], BMP9 was found to effectively activate Smads signaling, leading to an increased level of phosphorylated Smad1/5/8 (Fig. 1A). What is most noteworthy, however, is that exposure of C3H10T1/2 cells to BMP9 effectively increased the levels of phosphorylated p38 and ERK1/2, without altering the total amounts of these proteins. Similar results were also obtained in MEFs (Fig. 1B) and C2C12 cells (Fig. 1C). Furthermore, we also tested the effects of BMP9-conditioned medium (BMP9-CM) on activation of p38 and ERK1/2 in C3H10T1/2 cells. As illustrated in Fig. 1D, an increased level of phosphorylated p38 was first observed at 5 min, with its summit at 30 min post BM9-CM treatment. Similarly, the level of phosphorylated ERK1/2 was also increased, and peaked at 30 min. Collectively, these results strongly suggest that BMP9 can effectively promote activation of p38 and ERK1/2 MAPKs in MPCs. However, the exact functional roles of p38 and ERK1/2 in BMP9-induced osteogenic differentiation of MPCs need to be precise investigated.

**Figure 1:** BMP9 induces phosphorylation/activation of p38 and ERK1/2 in MPCs. (**A**). Western blotting analysis of BMP9-induced phosphorylation of Samd1/5/8, p38 and ERK1/2 in C3H10T1/2 cells. C3H10T1/2 cells were infected with Ad-BMP9 or Ad-GFP (MOI = 5), at 24 hrs, total amount and phosphorylated forms of Smad1/5/8, p38 and ERK1/2 was analyzed by western blotting. β-actin was used to demonstrate equal loading of all samples. (**B**) Western blotting analysis of BMP9-induced phosphorylation of p38 and ERK1/2 in MEFs. MEFs were infected with Ad-BMP9 or Ad-GFP (MOI = 5), at 24 hrs, total amount and phosphorylated forms of p38 and ERK1/2 was analyzed by western blotting. (**C**) Western blotting analysis of BMP9-induced phosphorylation of p38 and ERK1/2 in C2C12 cells. C2C12 cell were infected with Ad-BMP9 or Ad-GFP (MOI = 5), at 24 hrs, total amount and phosphorylated forms of p38 and ERK1/2 was analyzed by western blotting. (**D**) Western blotting analysis of BMP9 conditioned medium (BMP9-CM)-induced phosphorylation of p38 and ERK1/2 in C3H10T1/2 cells. C3H10T1/2 cells were treated with BMP9-CM, total amount and phosphorylated forms of p38 and ERK1/2 was analyzed at indicated time points by western blotting.

### BMP9-induced Early Osteogenic Differentiation of MPCs is Dramatically Blocked by the p38 Inhibitor, SB203580, but is Enhanced by the ERK1/2 Inhibitor, PD98059

To inspect the detail roles of p38 and ERK1/2 in BMP9-induced osteogenic differentiation of MPCs. C3H10T1/2 cells were exposed to BMP9 in the presence of SB203580 and PD98059, which are specific inhibitor of p38 and ERK1/2 respectively. Then, ALP activity was determined using chemiluminescence quantitative assay. By treating C3H10T1/2 cells with varying concentrations of SB203580 (0, 2, 5 and 10 µM), we found that SB203580 was able to significantly inhibit BMP9-induced ALP activity in a dose-dependent manner (Fig. 2A). Conversely, PD98059 (0, 10, 25 and 50 µM) treatment was found to remarkably enhance BMP9-induced ALP activity mostly in a dose-dependent manner (Fig. 2B). We also found similar effects of SB203580 and PD98059 on BMP9-induced ALP activity in MEFs (Fig. 2C) and C2C12 MPCs (Fig. 2D). These results strongly suggest us that p38 and EKR1/2 may exhibit opposing roles in regulating BMP9-induced early osteogenic differentiation of MPCs.

**Figure 2:** Opposing effects of p38 and ERK1/2 on BMP9-induced ALP activity of MPCs. (**A**) Inhibition of BMP9-induced ALP activity by p38 inhibitor SB203580 in C3H10T1/2 cells. C3H10T1/2 cells were infected with Ad-BMP9 or Ad-GFP (MOI = 5), followed by treatment with varying concentrations (0, 2, 5 and 10 µM) of SB203580. ALP activity was quantitative measured at day 7. Each assay condition was carried out in triplicate in at least two independent batches. “**”, p<0.01 (*vs*. control groups); “*”, p<0.05 (*vs*. control groups). (**B**) Enhancement of BMP9-induced ALP activity by ERK1/2 inhibitor PD98059 in C3H10T1/2 cells. C3H10T1/2 cells were infected with Ad-BMP9 or Ad-GFP (MOI = 5), followed by treatment with varying concentrations (0, 10, 25 and 50 µM) of PD98059. ALP activity was quantitative measured at 7 days. Each assay condition was carried out in triplicate in at least two independent batches. “**”, p<0.01; “*”, p<0.05 (*vs*. control groups). (**C**) Opposing effects of SB203580 and PD98059 on BMP9-induced ALP activity in MEFs. MEFs were infected with Ad-BMP9 or Ad-GFP (MOI = 5), followed by treatment with fixed concentrations of SB203580 (25 µM) or PD98059 (10 µM). ALP activity was quantitative measured at 5 days. Each assay condition was carried out in triplicate in at least two independent batches. “**”, p<0.01 (*vs*. control groups). (**D**) Opposing effects of SB203580 and PD98059 on BMP9-induced ALP activity in C2C12 cells. C2C12 cells were infected with Ad-BMP9 or Ad-GFP (MOI = 5), followed by treatment with fixed concentrations of SB203580 (25 µM) or PD98059 (10 µM). ALP activity was quantitative measured at 3 days. Each assay condition was carried out in triplicate in at least two independent batches. “**”, p<0.01 (*vs*. control groups).

As p38 and ERK1/2 are involved in regulating both cell proliferation and differentiation [52], [54], we thought that the opposing effects of p38 and ERK1/2 on BMP9-induced ALP activity of MPCs may partly correlate with the change of cell proliferation. Therefore, C3H10T1/2 cells were treated with BMP9 in the presence of SB203580 and PD98059 respectively, then ALP activity and cell proliferation was detected at selected time points. As illustrated in Fig. 3A and Fig. 3B, inhibition of ALP activity with SB203580 was accompanied by a lower level of cell proliferation, whereas PD98059 treatment led to a marked increase both in ALP activity and cell proliferation. Together, these findings indicate that the opposing effects of p38 and ERK1/2 on BMP9-induced ALP activity are partly in line with the change of cell proliferation.

**Figure 3:** Opposing effects of p38 and ERK1/2 on BMP9-induced ALP activity is correlated with the change of cell proliferation. (**A**) Effect SB203580 and PD98059 on BMP9-induced ALP activity in C3H10T1/2 cells. Subconfluent C3H10T1/2 cells were infected with Ad-BMP9 (MOI = 5) or Ad-GFP (MOI = 5), followed by treatment with SB203580 (25 µM) or PD98059 (10 µM), ALP activity was quantitative measured at the indicated time points. Each assay condition was carried out in triplicate in at least two independent batches. (**B**) Effect of SB203580 and PD98059 on BMP9-induced cell proliferation in C3H10T1/2 cells. Subconfluent C3H10T1/2 cells were infected with Ad-BMP9 (MOI = 5) or Ad-GFP (MOI = 5), followed by treatment with SB203580 (25 µM) or PD98059 (10 µM), cell proliferation was monitored by MTT assay at the indicated time points. Each assay condition was carried out in triplicate in at least two independent batches.

### Opposing Effects of p38 and ERK1/2 on BMP9-induced Late Osteogenic Differentiation of MPCs

Although ALP is a well-established early osteogenic marker, it is hardly an accurate predictor of the late stage of osteogenic differentiation and bone formation [11], [22], [23]. Thus, we sought to determine if p38 and ERK1/2 have any opposing effects on BMP9-induced late osteogenic markers, such as matrix mineralization and osteocalcin (OC) expression. We infected C3H10T1/2 cells and MEFs with Ad-BMP9 or Ad-GFP and then treated with SB203580 (10 mM) or PD98059 (25 mM). At 21 days post BMP9 treatment, Alizarin Red S staining was conducted to judge the effects of p38 and ERK1/2 on BMP9-induced matrix mineralization. Interestingly, SB203580 treatment deceased BMP9-induced matrix mineralization, on the contrary, PD98059 treatment increased matrix mineralization in C3H10T1/2 cells and MEFs (Fig. 4A). Next, we infected C3H10T1/2 cells with Ad-BMP9 in the presence of SB203580 or PD98059. At 9 days and 11 days post infection, total RNA was isolated from the cells for qPCR analysis. Likewise, we found that SB203580 resulted in a significant decrease in BMP9-induced OC expression. However, treatment by PD98059 led to a dramatically increase in BMP9-indcued OC expression at gene level (Fig. 4B). Moreover, we utilized immunocytochemical stain and further confirmed that BMP9-induced OC expression was inhibited by SB203580, and yet was enhanced by PD98059 at protein level (Fig. 4C). Taken together, the above results intensively suggest us that p38 and ERK1/2 may play important but opposing roles in regulating both early and late stages of BMP9-induced osteogenic differentiation of MPCs.

**Figure 4:** Opposing effects of p38 and ERK1/2 on BMP9-induced late osteogenic differentiation and Runx2 activation in MPCs. (**A**) Opposing effects of p38 and ERK1/2 on BMP9-induced matrix mineralization of MPCs. C3H10T1/2 cells and MEFs were infected with Ad-BMP9 or Ad-GFP, and then treated with SB203580 (25 mM) or PD98059 (10 mM). At day 21, cells were subjected to Alizarin Red S staining. Magnification, ×200. (**B**) qPCR analysis of SB203580 and PD98059 on BMP9-induced osteocalcin expression at gene level. C3H10T1/2 cells were infected with Ad-BMP9 or Ad-GFP, and then treated with SB203580 (25 mM) or PD98059 (10 mM). At day 9 and day 11, osteocalcin expression was detected by qPCR. All samples were normalized using endogenous levels of β-actin. “**”, p<0.01 (*vs*. control groups). (**C**) Immunocytochemical staining analysis of SB203580 and PD98059 on BMP9-induced osteocalcin expression at protein level. C3H10T1/2 cells were infected with Ad-BMP9 or Ad-GFP (MOI = 5), and then treated with SB203580 (25 mM) or PD98059 (10 mM). At day 12, cells were fixed and subjected to immunocytochemical staining analysis. Magnification, ×200. (**D**) Opposing effects of p38 and ERK1/2 on BMP9-induced Runx2 transcriptional activity. C3H10T1/2 cells were transfected with OC promoter containing Runx2-responsive element reporter, p6xOSE-Luc. Next, cells were infected with Ad-BMP9 in the presence of SB203580 (25 mM) or PD98059 (10 mM). At 36 hrs post infection, cells were lyzed for luciferase activity assay. Each assay condition was carried out in triplicate in at least two independent batches. Luciferase activity was normalized by total cellular protein concentrations among the samples. “**”, p<0.01 (*vs*. control groups). (**E**) qPCR analysis of SB203580 and PD98059 on BMP9-induced Runx2 expression at gene level. C3H10T1/2 cells were infected with Ad-BMP9 or Ad-GFP, and then treated with SB203580 (25 mM) or PD98059 (10 mM). At 24 and 48 hrs post treatment, Runx2 gene expression was detected by qPCR. Each assay condition was carried out in triplicate. All samples were normalized by endogenous level of β-actin. “**”, p<0.01 (*vs*. control groups). (**F**) Western blotting analysis of SB203580 and PD98059 on BMP9-induced Runx2 expression at protein level. C3H10T1/2 cells were infected with Ad-BMP9 or Ad-GFP, and then treated with SB203580 (25 mM) or PD98059 (10 mM). At 48 hrs post treatment, Runx2 protein expression was detected by western blotting. β-actin was used to demonstrate equal loading of all samples.

### Opposing Effects of p38 and ERK1/2 on BMP9-induced Runx2 Activation in MPCs

Runt-related transcription factor 2 (Runx2), also known as core-binding factor subunit alpha-1 (CBFα-1), is a key transcription factor associated with osteogenesis [55], [56]. Runx2 can directly stimulate expression of most of the well-established osteogenic markers, including osteocalcin (OC) [55]. It has been reported in our previous studies that Runx2 is a target of BMP9 [11], [20]. Therefore, we asked whether BMP9-induced activation of Runx2 was also influenced by p38 and ERK1/2 in an opposing model. Using a commonly used Runx2-regulated OC promoter reporter (p6xOSE-luc), we found that SB203580 treatment was able to inhibit BMP9-induced luciferase activity of p6xOSE-luc reporter, which contains Runx2-responsive elements and reflects Runx2 transcriptional activity. Conversely, PD98059 treatment increased BMP9-induced p6xOSE-luc reporter activity (Fig. 4D). These findings imply us that the effects of p38 and ERK1/2 on BMP9-induced Runx2 transcriptional activity are possibly opposing. Next, we examined the Runx2 expression at gene and protein level using qPCR and western blotting. As shown in Fig. 4E and Fig. 4F, BMP9-induced Runx2 expression was reduced by SB203580 treatment, and yet enhanced by PD98059 treatment at both gene and protein level. These results further confirm that p38 and ERK1/2 can exhibit opposing effects on BMP9-induced activation of Runx2 in an opposing manner. Token together, these above data reveal that p38 and ERK1/2 MAPKs are highly probably to play opposing roles in regulating BMP9-induced osteogenic differentiation of MPCs.

### Block of p38 and ERK1/2 Activity Leads to Opposing Effects on BMP9-induced Activation of Smads Signaling

We next sought to explore the possible mechanism behind the opposing effects of p38 and ERK1/2 on BMP9-induced osteogenic differentiation of MPCs. Smad1, 5, and 8 (Smad1/5/8) are classic mediators for BMPs osteoinductive signaling. It has been reported that candidate phosphorylated sites for MAPKs are existed in Smad1/5/8 proteins [57]. Moreover, MAPKs activation by BMPs has shown to influence Smads signaling in different cell models [9], [10], [26], [39]. Fig. 1A has confirmed that BMP9 was able to simultaneously induce activation of Smad1/5/8, p38 and ERK1/2. Therefore, we asked whether BMP9-activated Smads signaling was also changed in the presence of SB203580 or PD98059, respectively. Firstly, we examined the effects of SB203580 and PD98059 on phosphorylation of Smad1/5/8, the activated mediator of BMPs signaling. Upon BMP9 stimulation, phosphorylated Smad1/5/8 was increased and was effectively inhibited by SB203580. However, BMP9-induced phosphorylation of Smad1/5/8 was further enhanced by PD98059 (Fig. 5A). As BMP9-induced Smad1/5/8 phosphorylation was changed, we therefore postulated that the change of Smad1/5/8 phosphorylation ought to result in alternated nuclear translocation of these proteins. Using immunofluorescence stain, we found that SB203580 interestingly disrupted translocation of Smad1/5/8 to the nucleus. Conversely, PD98059 treatment enhanced BMP9-induced nuclear translocation of Smad1/5/8 (Fig. 5B). Lastly, we examined the ability of SB203580 and PD98059 on BMP9-induced transcriptional activity of Smad1/5/8. Using the BMPs responsive Smads reporter, p12xSBE-luc [22], [23], we found that SB203580 was able to neutralize BMP9-induced transcriptional activity of Smad1/5/8, however, PD98059 was capable of augmenting BMP9-induced Smad1/5/8 transcriptional activity (Fig. 5C). To sum up, inhibition of p38 and ERK1/2 activity led to opposing effects on BMP9-induced phosphorylation of Smad1/5/8, as well as its translocation to the nucleus, and subsequently transcriptional activity of Smad1/5/8. These above results imply us that p38 and ERK1/2 are likely to play opposing roles in regulating BMP9-induced osteogenic differentiation of MPCs partly through influence on Smads signaling cascade.

**Figure 5:** Inhibition of p38 and ERK1/2 activity leads to opposing effects on BMP9-indcued classical Smads signaling in MPCs. (**A**) Western blotting analysis of SB203580 and PD98059 on BMP9-induced Smad1/5/8 phosphorylation. Subconfluent C3H10T1/2 cells were pretreated with SB203580 (25 mM) or PD98059 (10 mM), and then treated with BMP9-CM. At 30 mins post BMP9-CM treatment, total amount and phosphorylated forms of Smad1/5/8 was analyzed by western blotting. (**B**) Immunofluorescence staining analysis of SB203580 and PD98059 on BMP9-induced nuclear translocation of Smad 1/5/8. Subconfluent C3H10T1/2 cells were pretreated with SB203580 (25 mM) or PD98059 (10 mM), and then treated with BMP9-CM. At 2 hrs post BMP9-CM treatment, nuclear translocation of Smad 1/5/8 by Immunofluenrescence staining. Magnification, ×200 (**C**) Luciferase reporter analysis of SB203580 and PD98059 on BMP9-induced Smad1/5/8 transcriptional activity. C3H10T1/2 cells were transfected with p12xSBE-luc. Next, cells were pretreated with SB203580 (25 mM) or PD98059 (10 mM), and then treated with BMP9-CM. At 36 hrs, cells were lyzed for luciferase activity assay. Luciferase activity was normalized by total cellular protein concentrations among the samples. “**”, p<0.01 (*vs*. control groups).

### Gene Silence of p38 and ERK1/2 Leads to Opposing Effects on BMP9-induced Osteogenic Differentiation of MPCs

Using specific inhibitors for p38 and ERK1/2 respectively, we found that p38 and ERK1/2 may exhibit opposing effects on BMP9-induced early and late osteogenic differentiation of MPCs through influence on classic Smads signaling cascade. To confirm that the effects of inhibitors were truly due to p38 and ERK1/2 inhibition and not a nonspecific drug effect, we employed adenoviruses expressing small interference RNA (siRNA) targeted p38 and ERK1/2 to infect C3H10T1/2 cells. Western blotting was carried out to assess the inhibitory efficiency of these siRNA on expressions of p38 and ERK1/2, respectively (Fig. 6A). Then, the effects of p38 and ERK1/2 knockdown on BMP9-induced osteogenic differentiation of MPCs were assessed. Similar to the results observed with SB203580, p38 knockdown was shown to inhibit BMP9-indcued ALP activity, as well as matrix mineralization and OC protein expression. In contrast, consistent with the data obtained from PD98059, ERK1/2 knockdown was found to enhance BMP9-induced ALP activity, matrix mineralization and OC protein expression (Fig. 6B, Fig. 6C, Fig. 6D). These results suggest that gene silence of p38 and ERK1/2 lead to opposing effects on BMP9-induced osteogenic differentiation of MPCs.

**Figure 6:** Knockdown of p38 and ERK1/2 leads to opposing effects on BMP9-indcued osteogenic differentiation of MPCs. (**A**) Effective knockdown of p38 and ERK1/2 expression by RNAi. C3H10T1/2 cells were infected with AdR-si-p38 or AdR-si-ERK1/2. At 24 hrs, total amount forms of p38 and ERK1/2 were analyzed by western blotting. NC, negative control. (**B**) Effect of p38 and ERK1/2 knockdown on BMP9-induced ALP activity. Subconfluent C3H10T1/2 cells were infected with AdR-si-p38 or AdR-si-ERK1/2, and then treated with BMP9-CM. ALP activity was quantitatively assessed at the indicated time points. “*”, p<0.05 (*vs*. control groups). (**C**) Effect of p38 and ERK1/2 knockdown on BMP9-induced matrix mineralization. C3H10T1/2 cells were Infected with AdR-si-p38 or AdR-si-ERK1/2, and then treated with BMP9-CM. At 21 days, cells were subjected to Alizarin Red S staining. Magnification, ×200. (**D**) Effect of p38 and ERK1/2 knockdown on BMP9-induced OC protein expression. C3H10T1/2 cells were infected with AdR-si-p38 or AdR-si-ERK1/2, and then treated with BMP9-CM. At day 12, cells were fixed and subjected to Immunocytochemical stain. Magnification, ×200. (**E**) Effect of p38 and ERK1/2 knockdown on BMP9-induced Smad1/5/8 phosphorylation. C3H10T1/2 cells were infected with AdR-si-p38 or AdR-si-ERK1/2, and then treated with BMP9-CM. At 30 min post BMP9-CM treatment, total amount and phosphorylated forms of Smad1/5/8 was analyzed by western blotting.

### Gene Silence of p38 and ERK1/2 Results in Opposing Effects on BMP9-induced Activation of Smads Pathway

We next sought to determine the influences of p38 and ERK1/2 knockdown on BMP9-induced Smad1/5/8 activity. Interestingly, BMP9-induced phosphorylation of Smad1/5/8 were accordingly decreased along with p38 RNAi, and yet increased along with ERK1/2 RNAi (Fig. 6E). Together, these results further confirm that p38 and ERK1/2 are likely to influence BMP9-induced Smads signaling cascade in a converse manner, through which to exert opposing effects on BMP9-induced osteogenic differentiation of MPCs.

### Opposing Effects of p38 and ERK1/2 on BMP9-induced New Bone Formation in Calvarial Organ Culture

The above *in vitro* data demonstrate that p38 and ERK1/2 may act in opposition to regulate osteoinductive activity of BMP9. To further investigate the regulatory roles of p38 and ERK1/2 on BMP9-induced bone formation, we conducted the calvarial organ culture experiments. Using calvariae of 4 days mouse pups, we found that treatment of BMP9 significantly stimulates new bone formation (in H&E staining, appeared as lighter color) over 7 days period [Fig. 7A and Fig. 7B]. It is noteworthy that inhibition of p38 activity by SB203580 led to a decrease in new bone formation compared with the BMP9 group, however, PD98059 treatment resulted in an increase in new bone formation (Fig. 7A and Fig. 7B). These results obtained from organ culture experiments suggest that p38 and ERK1/2 may act opposition to regulate BMP9-evokeed new bone formation.

**Figure 7:** Opposing effects of p38 and ERK1/2 on BMP9-induced new bone formation in calvarial organ culture. (**A**) Mouse calvariae was infected with Ad-BMP9, and then treated with SB203580 (25 µM) and PD98059 (10 µM). At 4 days post infection, calvariae was placed into fresh media and return to incubator for another 3 day until day 7. The amount of original bone remaining and new bone was assessed by H&E staining. Magnification, ×600. (**B**) measurement of new bone width using Image Pro Plus. “*”, p<0.05 (*vs.* BMP9).

### Gene Silence of p38 and ERK1/2 Results in Opposing Effects on BMP9-induced Ectopic Bone Formation in Subcutaneous MPCs Implantation *in vivo*

Lastly, we sought to confirm these above findings *in vivo* via MPCs implantation experiments. C3H10T1/2 cells were shown to be effectively co-infected with Ad-BMP9 and/or Ad-RFP, AdR-si-p38, AdR-si-ERK1/2 (Fig. 8A). The infected cells were collected and injected subcutaneously into athymic mice. At 5 weeks, the animals were euthanized, and the bony masses were retrieved (Fig. 8B). It seems that p38 knockdown did not affect the BMP9-transduced cells formed bony masses (Fig. 8C). However, ERK1/2 knockdown increased BMP9-transduced cells formed bony masses, which were noticeably bigger than those formed by the cells transduced by control groups (Fig. 8C). On histological evaluation, p38 gene silence inhibited BMP9-induced osteogenic differentiation and osteoblast maturation of C3H10T1/2 cells *in vivo*, with thinner trabeculae, more chondrocytes and a significant number of undifferentiated MPCs in H&E staining (Fig. 8D). Trichrome stain indicated that, while the BMP9 control samples exhibit abundantly fully ossified matrix, samples retrieved from p38 knockdown group display only focal ossification and a significant amount of cartilage matrix, implying immature osteogenesis (Fig. 8D). The presence of cartilage matrix in the samples co-infected with Ad-BMP9 and AdR-si-p38 was further confirmed by Alcian Blue stain (Fig. 8D). However, although ERK1/2 knockdown did not seem to affect BMP9-induced bone maturation, it was able to increase the quantity of bone formation, with more chicker trabeculae in H&E stain (Fig. 8D). Thus, in agreement with our *in vitro* studies, these *in vivo* results further substantiate the findings about the opposing roles of p38 and ERK1/2 in regulating BMP9-induced osteogenic differentiation of MPCs.

**Figure 8:** Knockdown of p38 and ERK1/2 leads to opposing effects on BMP9-indcued ectopic bone formation. (**A**) Co-infection efficiency of Ad-BMP9 and AdR-si-p38 (or AdR-si-ERK1/2). C3H10T1/2 cells were co-infected with Ad-BMP9 and AdR-si-p38 (or AdR-si-ERK1/2). At 24 hrs post co-infection, the co-infection efficiency was determined under a fluorescence microscope. (**B**) Macrographic images of ectopic bone mass. (**C**) Total volume of retrieved samples. “**”, p<0.01 (*vs.* control groups) (**D**) Histological stains of retrieved samples. Retrieved tissues were decalcified, fixed in 10% formalin overnight, and embedded in paraffin. Serial sections of the embedded specimens were stained with H&E, Masson’s Trichrome stain and Alcian Blue stain. BM, Bone Matrix; Ch, Chondrocyte; UMPCs, Undifferentiated mesenchymal progenitor cells; CM, Cartilage Matrix. Magnification, ×150.

## Discussion

BMP9 (also known as growth differentiation factor 2, or GDF2) was originally isolated from fetal mouse liver cDNA libraries and is a potent stimulant of hepatocyte proliferation [58]. Other roles of BMP9 include inducing the cholinergic phenotype of embryonic basal forebrain cholinergic neurons [59], regulating glucose and lipid metabolism in liver [60], and maintaining homeostasis of iron metabolism [61]. BMP9 is also a potent synergistic factor for murine hemopoietic progenitor cell generation and colony formation in serum-free cultures [62]. In previous studies, BMP9 has been proved to be most highly capable of inducing osteogenic differentiation of MPCs [11], [19], [20], [21]. Yet BMP9 remains as one of the least studied BMPs, and little is known about detail molecular mechanism underlying the BMP9-induced osteogenic differentiation of MPCs. Therefore, we are particularly interested in illuminating downstream signaling pathway(s) involved in BMP9 osteoinductive activity.

In this report, we investigate the detail roles of p38 and ERK1/2 MAPKs in BMP9-induced osteogenic differentiation of MPCs. We find that BMP9 simultaneously stimulates phosphorylation/activation of p38 and ERK1/2 in the osteogenic differentiation process of MPCs. BMP9-induced early and late osteogenic differentiation is decreased by p38 inhibitor SB203580, yet enhanced by ERK1/2 inhibitor PD98059. SB203580 is shown to inhibit BMP9-induced Runx2 activation, and to disrupt BMP9-activated Smads signaling. On the contrary, PD98059 treatment promotes BMP9-induced Runx2 activation and enhances BMP9-evokeed Smads signaling. The effects of inhibitors were reproduced with adenoviruses expressing siRNA targeted p38 and ERK1/2, respectively. We find that p38 and ERK1/2 act in opposition to regulate BMP9-induced new bone formation of cultured mouse calvarial organ. MPCs implantation studies also reveal that knockdown of p38 significantly decreases trabecular bone and osteoid matrix formation. However, ERK1/2 gene silence led to robust of trabecular bone. Together, our results strongly suggest that p38 and ERK1/2 are likely to play opposing regulatory roles in BMP9-induced osteogenic differentiation of MPCs partly through affecting Smads signaling cascade.

The physiological functions of MAPKs (mainly p38, ERK1/2 and JNKs) in osteogenic differentiation and bone formation have been deeply investigated both *in vitro* and *in vivo* [41], [42], [63], [64], [65], [66], [67], [68], [69], [70]. However, the obtained results from *in vitro* studies are controversial, with some studies suggesting a stimulatory role of MAPKs in osteogenic differentiation and bone formation [63], [64], [65], [66], and others proposing that MAPKs is inhibitory [41], [42], [67], [68]. The conflicting results of *in vitro* studies emphasize the need to explore the role of the MAPKs in osteogenic differentiation and bone formation by *in vivo* assay. Ge *et al*., showed that ERK1/2 activation was capable of stimulating osteoblast differentiation and fetal skeletal development through a pathway involving Runx2 in mice [69]. Using a transgenic mice model, Greenblatt *et al*., evidenced that p38 functions to phosphorylate osteogenic master gene Runx2 and promotes skeletogenesis and bone homeostasis [70]. These *in vivo* studies affirmatively supported that p38 and ERK1/2 MAPKs are play positive roles in regulating osteogenic differentiation and bone formation. Although *in vitro* and *in vivo* studies about the precise roles of MAPKs in skeletal development didn’t lead to complete unanimity, it is well established that MAPKs plays a functional role in osteogenesis and bone metabolism.

Several growth factors have shown to trigger MAPKs in different cell models [27], [28], [29], [30], [37], [71], [72], [73], [74]. IGF-1 promoted phosphorylation of p38, ERK1/2 and JNKs, through which to induce expression of osterix in human mesenchymal stem cells [37]. In MC3T3-E1 preosteoblastic cells, FGF-2 stimulated Runx2 phosphorylation and osteocalcin expression via activation of MAPKs [71]. Also, In PA-JEB or PA-JEB/β4 keratinocytes, p38 and ERK1/2 phosphorylation was increased after EGF stimulation during mitotic cell rounding [72]. HGF promoted activation of ERK1/2 and p38, and subsequently induced proliferation of lung adenocarcinoma cell line H441 [73]. In addition, MAPKs can also be activated by BMPs stimulation [26], [27], [28], [29], [30], [31], [32], [33], [34], [35], [36], [37], [38], [39], [40], [41], [42], which represents an important mechanism for non-Smads pathway(s) of BMPs signaling. The activation of MAPKs by BMPs could lead to various effects depending on the cell context. For example, BMP4 induced hepatocellular differentiation of rat hepatic progenitor cell was mediated by increase in activation of ERK1/2 [27]. BMP2-activated p38 was found to participate in BMP2-induced commitment of C3H10T1/2 MPCs to the adipocyte lineage [28]. BMP2 increased ALP activity and matrix mineralization through phosphorylation of p38α in human dental pulp cells (HDPCs) [29]. Moreover, BMPs-induced activation of MAPKs was also found to be essential for other physiological and pathological process, such as chondrogenesis, retina regeneration, tumor angiogenesis and cancer cells metastasis [30], [31], [32], [33].

Although BMPs could regulate tooth, kidney, skin, hair, muscle, haematopoietic and neuronal development, and maintain the iron metabolism and vascular homeostasis, the most intensive characterized function of BMPs is to induce osteogenic differentiation and bone generation. It has been described by various studies that MAPKs can activated by BMPs [26], [27], [28], [29], [30], [31], [32], [33], [34], [35], [36], [37], [38], [39], [40], [41], [42]. However, the exact effects of MAPKs on BMPs-induced osteogenesis are diverse and disputable, depending on the extracellular stimuli, the type of MAPKs and context of specific cells. By now, the studies about BMPs-activated MAPKs on BMPs-induced osteogensis were mainly focus on BMP2, and theses studies did not reach on consensus. For example, BMP2 inducement increased ERK1/2 activity in C3H10T1/2 MPCs, whereas nonfunctional ERK1/2 partially eliminated BMP2-induced ALP activity [36]. Celil *el al*., reported that BMP2 mediates osterix expression via activation of p38 and JNKs in human mesenchymal stem cells [37]. A study by Guicheux *el al*., also showed that p38 and JNKs were activated in response to BMP2 treatment in MC3T3-E1 preosteoblastic cells and primary cultured osteoblastic cells, and evidenced that these MAPKs have positive roles in regulating BMP2-induced osteogenic differentiation [38]. A study using C2C12 cells indicated that BMP2 activates ERK1/2 and p38 to promoting osteoblastic differentiation [39]. These above studies agree on the notion that MAPKs (p38, ERK1/2 and JNKs) play positive roles in BMP2-induced osteogenic differentiation. However, other studies using C2C12 and MC3T3-E1 cells obtain opposite results, showing that MAPKs (p38 and JNKs) have a negative role in BMP2-indcued osteogenic differentiation [40], [41], [42]. All these experiments did not ascertain the exact roles of MAPKs in BMPs-induced osteogenesis because of the controversial results. However, it is convincingly supported that MAPKs play essential roles in regulating osteogenic activity of BMPs, with positive or negative effects.

In the current study, we examine the ability of BMP9 to activate p38 and ERK1/2 MAPKs, and the contribution of each MAPKs to regulate BMP9-induced osteogenic differentiation of MPCs. BMP9 was able to activate ERK1/2 and p38 MAPKs in MPCs. Importantly, inhibition of p38 and ERK1/2 activity led to opposing effects on BMP9-induced osteogenic differentiation of MPCs both *in vitro* and *in vivo*. Therefore, we conclude that p38 and ERK1/2 exert opposing influences on BMP9-induce osteogenic differentiation of MPCs. The notion that ERK1/2 and p38 act in opposition has been reported in various studies. FGF2 was able to simultaneously increase phsphorylation of ERK1/2 and p38, blocking of p38 activity promotes process extension whereas inhibition of ERK1/2 activity leads to reduce of process extension [74]. Oncogenic transformation by H-Ras was found to involve down-regulation of tropomyosin, which in turn depended on the simultaneously activation of ERK1/2 and inactivation of p38 MAP kinase [75]. Dipyrithione (2, 2′-dithiobispyridine-1, 1′-dioxide, PTS2), a pyrithione derivate, was shown to activate p38 and ERK1/2, suppression of p38 by SB203580 reduced the PTS2-induced apoptosis of the HeLa cells, whereas inhibition of ERK1/2 with PD98059 increased apoptosis [76]. P38 and ERK1/2 have also been reported to mediate BMP4-induced osteogensis of muscle-derived stem cells in an opposing manner [77]. Thus, the balance of ERK1/2 and p38 activities may be a key regulatory signal for many biological and pathophysiological responses, including BMP9-induced osteogenic differentiation of MPCs.

In conclusion, we find that BMP9 are shown to activate p38 and ERK1/2 in the induction of the osteogenic differentiation of MPCs, implying that p38 and ERK1/2 are essential regulatory components in BMP9 osteoinductive activity. Notably, using specific inhibitor and siRNA for p38 and ERK1/2 respectively, we find that p38 and ERK1/2 may act opposition to regulate BMP9-indcued early and late osteogenic differentiation of MPCs *in vitro*. Calvarial organ culture and subcutaneous MPCs implantation studies confirm the opposing effects of p38 and ERK1/2 on BMP9-indcued osteogenesis and bone formation *in vivo*. Furthermore, we explore the possible molecular mechanism involved, and find that p38 and ERK1/2 are likely to fulfill opposing regulatory effects on BMP9-indcued osteogenic differentiation of MPCs via exert influence on Smads signaling cascades. This knowledge will provide insights into the molecular mechanisms by which BMP9 induces osteogenic differentiation of MPCs. However, other signaling molecules possible involved also need to be intensive characterized and illustrated. Our unpublished data have shown that JNKs and ERK5 MAPKs are also activated in BMP9-induced osteogenic differentiation, implying other members of MAPKs are highly probably involved in regulating BMP9-induced osteogenesis and bone formation. Therefore, future studies should be devoted to the elucidation of detail cross-talk between diverse signal molecules (including JNKs and ERK5 MAPKs) in the context of BMP9-induced osteogenic differentiation of MPCs and bone formation.

## Supporting Information

Table S1 **Primers used in qPCR.**
(DOC)
